# Comparison of immunohistology using pan-CK and EMA in the diagnosis of lymph node metastasis of gastric cancer, particularly micrometastasis and isolated tumor cells

**DOI:** 10.3892/ol.2012.1078

**Published:** 2012-12-14

**Authors:** YI YANG, JUNWEI LI, SHANHUA MAO, HONGGUANG ZHU

**Affiliations:** 1 Departments of General Surgery, Shanghai Medical College, Fudan University, Shanghai 200032, P.R. China; 2 Obstetrics and Gynecology, Shanghai Medical College, Fudan University, Shanghai 200032, P.R. China; 3 Urology, Shanghai Medical College, Fudan University, Shanghai 200032, P.R. China; 4 Pathology, Shanghai Medical College, Fudan University, Shanghai 200032, P.R. China

**Keywords:** pan-cytokeratin, epithelial membrane antigen, metastasis, micrometastasis, isolated tumor cell

## Abstract

The aim of this study was to identify a suitable method for detecting lymph node metastasis of gastric cancer (GCA) by hematoxylin and eosin (HE) and immunohistochemical (IHC) staining. We investigated lymph node metastasis using pan-cytokeratin (CK) and epithelial membrane antigen (EMA) IHC staining in a total of 1,422 lymph nodes from 100 patients who underwent radical gastrectomy between 2007 and 2009. Of 700 intestinal and 722 diffuse type GCA lymph nodes, the metastasis rates were significantly different when using conventional HE staining only or HE supplemented with IHC (P<0.01). The metastasis rate of the intestinal type was 31.71% using HE staining, 35.71% with HE and pan-CK, 35.57% with HE and EMA and 35.71% with combination examinations of all three. The false-positive rate was zero with pan-CK, 12.67% with EMA and 18.57% with all three. The metastasis rate of the diffuse type was 27.70% using HE staining, 36.01% with HE and pan-CK, 35.04% with HE and EMA and 36.01% with all three. The false-positive rate was zero with pan-CK, 7.58% with EMA and 11.86% with all three. For both types, the true-positive and -negative rates of pan-CK were higher than those of EMA. IHC staining is unnecessary if lymph node metastasis is detected in HE staining. If HE staining does not reveal metastasis, pan-CK staining should be performed for further diagnosis.

## Introduction

According to WHO classification, gastric cancer (GCA) can be divided into two major categories, intestinal and diffuse types (1). Lymph node metastasis of GCA decides the tumor-node-metastasis (TNM) stage. Lymph node micrometastasis (MM) in GCA is also a significant prognostic factor and influences the therapeutic regimen (2–5), while isolated tumor cell (ITC) is a type of MM. In routine pathology practice, ×40 microscopy of hematoxylin and eosin (HE) staining is commonly used to detect lymph node metastasis. However, misdetection often occurs with this method.

In clinical practice, we also find that lymph node metastasis of intestinal type GCA is glandular-like and little misdetection occurs in HE staining; however, diffuse type GCA is the opposite. Cancer cells are isolated in the primary tumor and lymph node metastases, especially in MM/ITC. Misdetection occurs more often in conventional HE staining.

Certain studies have claimed that regular HE staining supplemented with immunohistochemistry [IHC; cytokeratin (CK) or epithelial membrane antigen (EMA)] may increase the detection rate of lymph node metastasis of GCA (6–8) by providing more accurate pathological information so as to guide treatment and prognosis prediction (9). However, of these studies, some used pan-CK as an independent indicator, some EMA and others a combination to detect the metastasis. We find that some non-epithelial cells, such as plasma cells, are positive, while some cancer cells are negative in EMA staining in our routine work. Therefore, the questions of which is the best marker for detecting the lymph node metastasis of GCA and whether the combination of CK and EMA increases the metastasis detection rate remain unsettled.

## Patients and methods

### Patients and specimens

Among the patients who underwent radical gastrectomy at the Department of Surgery at Hua Shan Hospital (tertiary referral center in China) between 2007 and 2009, 50 patients with intestinal type GCA and 50 with diffuse type GCA were reviewed. We collected 700 lymph nodes dissected from patients with intestinal type GCA and 722 from patients with the diffuse type. The mean age of this series of patients was 57.88±13.53 years (range, 28–81), while that of the intestinal type patients was 59.88±13.48 years and for the diffuse type was 55.45±13.32 years. The study was approved by the Ethics Committee of Huashan Hospital, Fudan University, Shanghai, China. Informed patient consent was obtained from all the patients.

### IHC staining

A total of 1,422 lymph nodes were resected from the 100 patients and a single pathologist reexamined all lymph node slides to confirm the absence of lymph node metastasis. IHC staining for CK and EMA was performed using the ABC IHC staining method. From paraffin blocks, the widest area that represented the condition of the corresponding lymph node was sectioned at 4-mm thickness, and the tissue sections were deparaffinized by immersion in xylene and rehydration in a series of alcohol. To augment the expression of antigen in tissues, citrate buffer solution was added to the samples which were then boiled in a microwave oven. To suppress the endogenous peroxidase activity, the samples were treated with 3% hydrogen peroxide solution for 15 min and rinsed with phosphate-buffered saline (PBS). To prevent non-specific immune reactions, the samples were reacted with normal horse serum for 20 min. The slides were shaken lightly and then reacted with primary antibody at 37°C for 90 min. A 1:100 dilution of mouse-anti-human broad-spectrum CK antibody AE1/AE3 (M-0349 200912) or a 1:200 dilution of mouse-anti-human EMA monoclonal antibody (M-0236 200912) was used as the primary antibody. After rinsing the slides with PBS, a 1:200 dilution of secondary antibody (VECTOR peroxidase mouse IgG PK-4002) was added and the mixture were reacted at 37°C for 60 min and then rinsed with PBS. Subsequently, ABC solution was added, reacted for 30 min and the samples were rinsed with PBS. DAB was then added, reacted for 5 min and the samples were rinsed with the buffer solution, counter-stained with Mayer’s hematoxylin and sealed with resin mount (060440303018 Leica LV Ultra). The negative control was prepared by the same procedure with lymphoid follicles of the amygdala and tonsil epithelia were used as the positive control.

### Evaluation of staining results

CK is located in the cytoplasm (10) and EMA on the cell membrane (11,12). Positive staining cells are brown-yellow, while the negative cells are unstained. Positive staining lymph nodes were confirmed by examination of the structure and morphology of the cells.

If IHC-positive cancer cells were detected in the lymph node as a single cell or a small nest of cancer cells <0.2 mm in size, it was defined as ITC. If the size of the cell nest was >0.2 mm but <2 mm, it was defined as MM. However, MM and ITC were combined into one group in the subsequent statistical analysis as there were few cases of ITC in our study (13). Two senior pathologists independently observed the HE, CK and EMA staining slides under a microscope to determine the results. For the HE-, CK- and EMA-positive staining slides, ×100 microscopy of the HE sections was used to determine whether the positive IHC results were tumor metastasis. A single pathologist reexamined all slides to confirm the absence of lymph node metastasis.

### Statistical analysis

For comparison of the detection rate of CK and EMA staining method, we calculated the detection, true-positive, true-negative and false-positive rates. Statistical comparisons were performed using a four-fold table and a paired marginal χ^2^ test, Fisher’s exact probability and Student’s t-test. P<0.05 was considered to indicate a statistically significant result. The statistical analysis software SPSS 15.0 was used (SPSS, Inc., Chicago, IL, USA).

## Results

### Detection rate of lymph node metastasis

A total of 1,422 lymph nodes were resected from the 100 patients (50 intestinal GCA and 50 diffuse GCA). Of those lymph nodes, 700 were dissected from intestinal type GCA and 722 from diffuse type. Of the patients with intestinal type GCA, 222/700 were node-positive, with a detection rate of 31.71%, while in the diffuse type, 200/722 were node-positive, with a detection rate of 27.70%, by conventional HE staining. Following examination by both HE and IHC staining, 250/700 (35.71%) intestinal cases and 260/722 (36.01%) diffuse cases were node-positive. A total of 28 intestinal type and 60 diffuse type lymph nodes were found to be positive by IHC staining which were missed by HE staining. All these foci were found to be MM/ITC.

### CK IHC staining

In intestinal and diffuse type GCA, 250 and 260 lymph nodes were positive for metastasis by CK staining and the detection rate increased from 31.71% to 35.71% (P<0.01) and from 27.70% to 36.01% (P<0.01), respectively (Table I). Therefore, there was misdetection by HE staining (Fig. 1).

There was no false-positive or false-negative case of CK staining in the two types of GCA following confirmation under ×100 microscopy (Table II).

Among EMA-negative lymph nodes, one intestinal type and seven diffuse type lymph nodes were positive by both CK and HE staining. However, there were no cases of EMA-positive tumor cells which were negative by CK staining (Table II; Fig. 2).

### EMA IHC staining

In intestinal type and diffuse type, 306 and 288 lymph nodes were positive for metastasis by EMA staining, while the detection rate increased by 37.84% and 44.00%, respectively (P<0.01; Table I).

One of the 250 intestinal type lymph nodes was negative by EMA staining but contained cancer cells when viewed under ×100 microscopy. Of the diffuse type cases, seven out of 260 lymph nodes were negative. The false-negative rates were 0.40% and 2.69%, respectively (Table II).

In certain cases, normal cells were positive by EMA staining. A total of 57 out of 450 intestinal type and 35 of 462 diffuse type lymph nodes were false-positive. These false-positive foci were mostly germinal centers and plasma cells (Fig. 3).

### Combination of CK and EMA IHC staining

In the two types of GCA, the combined use of HE and IHC staining did not increase the detection rate of lymph node metastasis and increased the false-positive rate.

Among the intestinal type cases, the true-positive rate of CK staining was higher than that of EMA staining (100 and 99.60%, respectively), as was the true-negative rate (100 and 97.31%, respectively; Table II).

Among the diffuse type cases, the true-positive rate of CK staining was also higher than that of EMA staining (100 and 97.31%, respectively), as was the true-negative rate (100 and 92.42%, respectively; Table II).

## Discussion

Lymph node metastasis can be divided into three types, including macrometastasis, MM and ITC. Presently, GCA is one of the most malignant tumors while lymph node MM/ITC always occurs in the early stage. Lymph node MM plays a main role in stage confirmation, prognosis and the selection of clinical therapeutic regimen. MM/ITC exists in up to 30% of HE-negative lymph nodes (13,14). There have been several studies evaluating the correlation between MM/ITC and prognosis in GCA (2,15–17). Most studies reported that MM/ITC affected the prognosis of GCA, but the degree of influence was variable according to the groups of patients. One study reported that both CK and EMA staining increased the sensitivity and specificity of the detection rate of lymph node MM/ITC and decreased the rate of misdetection. pan-CK (AE1/AE3) and EMA are epithelium-specific antibodies. As the basic component of cellular structure of normal epithelial cells and epithelial cancer cells, they are often used to differentiate tumors according to whether they originate from the epithelium or not. However, no study has confirmed which of CK and EMA is the better method for raising the detection rate of lymph node MM/ITC, and whether it is necessary to perform combined CK and EMA examinations. Our study demonstrates that IHC staining increases the detection rate of lymph node metastasis. All the misdetected foci of metastasis were confirmed to be MM/ITC.

CK staining is valuable in assisting diagnosis and selecting a suitable clinical treatment. Some HE-negative slides were CK-positive due to MM/ITC. There were significant differences between HE and CK staining when the cases were checked under ×40 light microscopy. There was no false-positive or false-negative case of CK staining in either type of GCA, as confirmed under ×100 microscopy.

Although there are differences between the results of EMA and HE staining, false-positive and false-negative rates of EMA staining are much higher. The reasons for this are as follows. Firstly, some HE-positive slides were EMA-negative and MM/ITC is more easily missed in EMA staining. Secondly, HE-negative slides were EMA-positive. The visual field of EMA staining is not as clear-cut as in CK staining (18,19). Inexperienced pathologists may falsely regard this non-specific staining as positive and make a false diagnosis. Thirdly, the germinal centers of lymph nodes appear to be positive. Certain studies have reported that germinal centers may be false-positive under EMA staining in patients with T lymph cell lymphoma. Fourthly, plasma cells may also be stained. Some authors also report that plasma cells may be false-positive in EMA staining, characterized as the focus of MM/ITC of the diffuse type GCA, which may lead to misdiagnosis (20,21).

It is unnecessary to perform combined CK and EMA examinations to detect the lymph node metastasis of GCA. It may increase the false-positive rate, but is unlikely to improve the detection rate.

The present study has certain limitations. Although CK staining increases the detection rate of lymph node metastasis of GCA, MM/ITC appears as only a single cell or a small nest of cancer cells. This means that the focus will not occur in all the slides of one paraffin block, which may cause misdetection in IHC or HE staining.

There is no need to perform EMA examination, due to the false-positive and false-negative situation. For the two types of GCA, CK should be used to confirm whether MM/ITC exists if conventional pathology is negative. Since the focus of lymph node MM/ITC appears as isolated cells or a small nest of cancer cells, it may be easily missed in HE staining only. However, HE staining is sufficient if the lymph node is positive under routine pathological examination.

Our research compares the methods of HE, CK and EMA staining, aiming to demonstrate the work process of diagnosing lymph node metastasis, especially MM/ITC, of GCA.

## Figures and Tables

**Figure 1:** HE misdetection. (A) pan-CK staining of a lymph node shows several isolated tumor cells (×40). (B) EMA staining of the corresponding lymph node shows several isolated tumor cells (×40). (C) HE staining of the corresponding lymph node shows no clearly visible tumor cells in the lymph node (×40). HE, hematoxylin and eosin; pan-CK, pan-cytokeratin; EMA, epithelial membrane antigen. Arrows indicate isolated tumor cells.

**Figure 2:** EMA misdetection. (A) CK staining of a lymph node shows a patch of tumor cells (arrow) (×40). (B) EMA staining of the corresponding lymph node shows no clearly visible tumor cells in the lymph node (arrow) (×40). (C) HE staining of the corresponding lymph node shows a patch of tumor cells (arrow) (×40). (D) ×100 microscopy of HE slides of the corresponding lymph node proves to be tumor cells. CK, cytokeratin; EMA, epithelial membrane antigen; HE, hematoxylin and eosin.

**Figure 3:** False-positive EMA staining. Upper panel shows germinal centers (indicated by arrows). (Aa) pan-CK staining of germinal centers in a lymph node shows non-tumor cells. (Ab) EMA staining of germinal centers in the corresponding lymph node shows a patch of tumor cells. (Ac) ×40 microscopy of HE slides of the corresponding lymph node proves to be non-tumor cells. Lower panel shows plasma cells (indicated by arrows). (Ba) pan-CK staining of plasma cells in a lymph node shows non-tumor cells. (Bb) EMA staining of plasma cells in the corresponding lymph node shows a patch of tumor cells. (Bc) ×100 microscopy of HE slides of the corresponding lymph node proves to be non-tumor cells. EMA, epithelial membrane antigen; pan-CK, pan-cytokeratin; HE, hematoxylin and eosin.

**Table I:** Chi-square analysis of detection rate of pan-CK, EMA and HE (×40).

	HE (×40)				
Sample	(+)	(−)	Total	Chi-square	P-value
Intestinal					
pan-CK					
(+)	222	28	250	28.00	<0.01
(−)	0	450	450		
Total	222	478	700		
EMA					
(+)	221	85	306	82.05	<0.01
(−)	1	393	394		
Total	222	478	700		
Diffuse					
pan-CK					
(+)	200	60	260	600.00	<0.01
(−)	0	462	462		
Total	200	522	722		
EMA					
(+)	193	95	288	75.92	<0.01
(−)	7	427	434		
Total	200	522	722		

HE, hematoxylin and eosin; pan-CK, pan-cytokeratin; EMA, epithelial membrane antigen.

**Table II:** Comparison of true-positive and true-negative rates of CK and EMA.

Sample	HE ×100 (+)	HE ×100 (−)	True-positive rate (%)	True-negative rate (%)
Intestinal				
pan-CK (+)	250	0	100	100
pan-CK (−)	0	450		
EMA (+)	249	57	99.60	87.33
EMA (−)	1	393		
Diffuse				
pan-CK (+)	260	0	100	100
pan-CK (−)	0	462		
EMA (+)	253	35	97.31	92.42
EMA (−)	7	427		

CK, cytokeratin; EMA, epithelial membrane antigen; HE, hematoxylin and eosin.
